# Finite Element Analysis of Femoral-Acetabular Impingement (FAI) Based on Three-Dimensional Reconstruction

**DOI:** 10.1155/2022/2937056

**Published:** 2022-02-27

**Authors:** Xi Luo, Jun Zhang, Guofeng Cai, Yuqiong Wu, Kun Ma

**Affiliations:** ^1^College of Architectural Engineering, Kunming University of Science and Technology, Kunming 650500, Yunnan, China; ^2^Department of Orthopedics, Second Affiliated Hospital of Kunming Medical University, Kunming 651000, Yunnan, China; ^3^Department of Sports Medicine, First Affiliated Hospital of Kunming Medical University, Kunming 651000, Yunnan, China

## Abstract

In order to solve the problem that people often have pain in the hip joint, it is more meaningful to study femoral-acetabular impingement syndrome in the future. This article aims to study the finite element analysis of femoral-acetabular impingement based on three-dimensional reconstruction. This paper proposes a selective image matching strategy. In the feature matching stage, all images are not matched in pairs, but the corresponding camera distance between the images is calculated initially, which has little effect on the number of features and greatly reduces the time of feature matching, thereby reducing the time cost of 3D reconstruction. In this experiment, a double-blind experiment was used to check the range of motion of all hip joints. Two senior radiologists read the obtained hip joint orthographic films to screen out the hip joint orthographic films that meet the requirements. Experimental data shows that although the initial matching points of the algorithm in this paper are lower than those of the traditional algorithm, the final number of matching points is higher than that of the traditional algorithm. When the final number of patches is fixed to 10000, the initial patch required by the algorithm in this paper is more than that required by the SAD algorithm, nearly 13%, but the total storage requirement is 56.4% of the SAD algorithm, which is a big improvement.

## 1. Introduction

With the rapid development of computer technology and multimedia technology, signal and image processing technology has received more and more attention. Three-dimensional object and environment reconstruction, as an important branch, has attracted the attention of a large number of scholars at home and abroad and obtained greater progress and a lot of results. Generally speaking, three-dimensional reconstruction is to use existing algorithms or related three-dimensional reconstruction software to model the object or environment, so as to obtain the three-dimensional model that people want.

Among the various ways the human body perceives the external world, vision is the most direct way. In all perceptions of the external world, most of the information comes from vision. Machine vision is based on the perception system that simulates the human eye, so that computers or related machines can obtain and recognize two-dimensional images, so that they have the ability to perform a series of tasks such as three-dimensional positioning, three-dimensional drawing, and three-dimensional reconstruction. On this basis, the extended stereo vision uses images and videos taken by cameras to realize the cognition of the objective world and uses robots to detect areas that cannot be reached by humans or areas that are more dangerous. Shoot to build a three-dimensional model of this type of environment or object. The development of computer vision has promoted human cognition of the unknown world and led to the development of medicine. Because of the abnormal anatomical morphology of the femur and acetabulum, the abnormal collision of the proximal femur and acetabular margin occurs at the end of hip movement. It occurs in young people who exercise a lot and is prone to early hip degeneration.

Parth used two large-capacity hip sparing centers to retrospectively review the hip sparing database of staged bilateral hip arthroscopy from 2008 to 2015 and determine the degree of correlation of imaging measurements, the degree of correlation of intraoperative pathology, and the difference in results on both sides of patients who need to stage bilateral hip arthroscopy [1]. Xie Z believed that femoral-acetabular impingement is a common hip joint disease that may make many patients weak. Hip arthroscopy is used to treat impinging CAM and clamp-shaped acetabular lesions. In view of the low cost of 3D hip printing, no radiation exposure, and tactile multi-angle views, he proposed a safer and more repeatable intraoperative technique than traditional fluoroscopy to achieve better results after femoral-acetabular impact surgery the resection and results [2]. Dutra B believed that in the past ten years arthroscopic treatment of hip joint diseases has been significantly spread and developed, and it currently represents the gold standard for the treatment of athletes' femoral-acetabular impingement. The function of the joint capsule has been better understood, sparking intense debate. He retrospectively included 36 patients (competitive athletes) who underwent hip arthroscopy for femoral-acetabular impingement for two years (2016–2018). It is concluded that the new longitudinal shape of the capsulotomy technique and the unilateral suture of the capsular suture at the end of the athlete's surgery can have a positive effect on the patient's functional outcome [3]. Lutter C analyzed the mechanical environment of the intra-articular structure of femoral-acetabular impingement syndrome, and further understood its pathomechanical characteristics. Based on CT data, a three-dimensional finite element mechanical analysis model of the hip joint including normal articular cartilage and femoral-acetabular impingement syndrome was accurately constructed [4]. Kemp J L reviewed patients who underwent hip arthroscopy at the Children's Hospital for idiopathic femoral-acetabular impingement or acetabular labrum tear and analyzed demographic predictors by using univariate logistic regression with generalized estimating equations. A matched case-control analysis was then performed to determine the radiological predictors of acetabular cartilage lesions by using univariate and multivariate conditional logistic regression. It was found that, in adolescents undergoing hip arthroscopy, older age, men, and higher body mass index were predictors of acetabular cartilage disease. From an imaging point of view, the increased *α* angle increases the possibility of acetabular cartilage disease, and the presence of the cross sign reduces this possibility. When considering hip arthroscopy to facilitate preoperative planning and more accurately set patient expectations, it is important to predict the presence of acetabular cartilage lesions [5, 6]. Angsutanasombat C believed that a single reconstruction of an object is very important in many applications, where the object is moving, or its shape is non-rigid and changes irregularly. He proposed a single-shot structured light 3D imaging technique, which calculates a phase map based on a distorted line pattern. This technology uses image processing technology to segment and cluster projected structured light patterns from a single captured image. The coordinates of the cluster lines are extracted to form a low-resolution phase matrix and then transformed into a full-resolution phase map by spline interpolation [7]. Vahedi H believed that Morgagni hernia (MH) can be diagnosed by different utilities, but all of these methods are not always 100% accurate. Three-dimensional (3D) reconstruction models help to better understand important anatomical structures. He reported a case of MH that had been misdiagnosed as diaphragmatic valgus in other institutions and provided laparoscopic repair based on the 3D reconstruction model. This case emphasizes that the 3D reconstruction model can be a useful supplementary tool for the diagnosis and preoperative evaluation of MH patients, especially when its diagnosis in clinical practice is confused [8].

The innovations of this article are as follows. (1) Using a double-blind experiment, two senior radiologists read the obtained hip joint orthographic film, and according to the PINCER-type FAI hip joint orthographic film imaging signs inclusion criteria and exclusion criteria, using a double-blind method to check the range of motion of all hip joints. Because machine learning is intelligent and the identified data is more accurate, we used machine learning to evaluate the femoral-acetabular impact finite element analysis. (2) The pathogenesis of FAI is the abnormal anatomical morphology of the hip joint. Three-dimensional reconstruction technology is used to perform imaging signs of the femoral-acetabular impingement. (3) Optimizing the selection of image pairs in the feature matching process, changing from the original full image matching to querying adjacent distance images for matching, which greatly reduces the time complexity and does not affect the quantity and quality of feature point matching. (4) The research on femoral-acetabular impingement is mainly applied to the treatment of femoral-acetabular impingement in the medical field and promotes the development of medicine in this field and makes new breakthroughs in the treatment of femur.

## 2. Finite Element Analysis Method of Femoral-Acetabular Impingement (FAI) Based on Three-Dimensional Reconstruction

### 2.1. Femoral-Acetabular Impingement Syndrome

#### 2.1.1. Basic Concepts

The current mainstream view of the disease believes that this so-called “impingement” is a common cause of hip pain in most young patients who have ruled out obvious organic hip disease and classifies it as hip osseous, one of the causes of arthritis [9]. Since the definition was proposed, a large number of scholars have conducted research on it from many directions and have made certain progress and have further in-depth understanding of the disease. According to the different manifestations of imaging, the disease is divided into three types: cam type (CAM-type), clamp type (PINCER-type), and mixed type (MIX type); it is believed that the disease should be diagnosed at an early stage and related treatment [10, 11]. However, with a large number of clinical observations, it has been found that the x-ray signs of the so-called FAI also have a large number of manifestations in people without any hip symptoms; a study by Laborie et al. found that about half of adults without hip symptoms have at least one or more FAI-related symptoms. X-ray imaging is abnormal. Hartofilakidis et al. conducted a long-term follow-up of 96 patients with FAI-related radiological abnormalities but asymptomatic. Among them, only 17 cases developed osteoarthritis after an average follow-up of 12 years, and the remaining 79 cases were followed up for an average of 18.5 years without bones and joints [12]. In this regard, many scholars have questioned the concept to a certain extent, questioning whether it has over-defined this so-called “impact” [13].

Femoral-acetabular impingement syndrome is a hip joint disease that has been proposed for more than a decade. The current mainstream view is that this so-called “impingement” causes most of the young patients who have ruled out obvious organic hip joint disease, the more common cause of hip pain, and it is listed as one of the causes of hip osteoarthritis [14]. Since this definition was proposed, a large number of scholars believe that the disease should be diagnosed and treated at an early stage. However, with a large number of clinical observations, it has been found that the so-called “impact” signs are also present in a large number of people without any hip symptoms. In this regard, many scholars have questioned the concept to a certain extent, questioning whether it has over-defined this so-called “impact” [15]. Checking the relevant domestic and foreign literature since the concept was put forward, there is no clear diagnosis standard and treatment indication for the disease at present.

#### 2.1.2. Cause

Strictly speaking, the cause of the disease has not yet been fully clarified. According to GANZ, the abnormal anatomy of the proximal femur and acetabulum is the basis of the disease [16]. This so-called abnormal anatomy will reduce the relative movement space of the femur and the acetabulum when the hip joint moves, resulting in abnormal contact. With the in-depth study of the disease, certain acquired factors will cause changes in the anatomical structure of the hip joint, which will also become the cause of FAI [17]. In addition, studies have shown that even if the anatomical structure of the hip joint does not have the above abnormal performance, when its range of motion exceeds the normal range, there will be “impact” between the proximal femur and the acetabular rim, which to some extent also confirms GANZ on the basis of the pathogenesis of the disease, that is, the theoretical view of the abnormal hip joint structure [18].

#### 2.1.3. Imaging Examination

Figure 1, shows an imaging examination of the hip joint. Currently, the most widely used initial diagnosis of FAI is the x-ray examination of the hip joint. The spatial distribution of anatomical structures obtained by plain radiographs is incomparable with CT and MRI, and it plays an irreplaceable role in structural diseases of bones and joints. The imaging diagnosis of FAI mainly relies on the measurement and evaluation of the hip joint anatomy on the plain film of the hip joint. The pelvic orthographic film has incomparable advantages in this respect. The premise is that the obtained hip joint orthographic film is a standard orthographic film. A more satisfactory orthographic film is that the longitudinal distance between the midpoint of the sacrococcygeal joint and the midpoint of the pubic symphysis is less than 3 cm, the lateral distance is less than 1.5 cm, and the pelvis has no obvious tilt. The obtained pelvic radiographs need to be measured for comprehensive evaluation. The most commonly used measurement items are CE angle, eccentricity, cross sign, head socket index, acetabular deep hip index, HTE angle, alpha angle, etc. [19, 20].

Compared with the spatial distribution of plain radiographs, CT scan of bone tissue has a higher spatial resolution, especially the reconstruction of three-dimensional CT, which can more intuitively observe the spatial structure of bones. A CT scan helps to analyze the shape of the acetabulum and femoral head, the eccentricity of the femoral head and neck, etc. On the CT cross section of the acetabulum, it can be observed whether there is excessive coverage of the anterior and posterior walls of the acetabulum. The anatomical morphology of the femoral head-neck junction can be clearly observed in the coronal view, and the presence of retroversion of the acetabulum can be identified in the sagittal view. Some of the main diagnostic indexes of FAI can be determined more accurately, such as femoral head-neck offset, *α* angle, so as to better assess the FAI classification and the degree of damage [21].

For early FAI pelvic plain film and CT, it is difficult to find bone changes, especially cartilage changes. MRI has obvious advantages [22]. As a non-invasive examination method, MRI can detect abnormal anatomical morphology of the femoral head and neck junction and excessive coverage of the acetabulum. It is currently the only method that can directly show the damage of the labrum and articular cartilage in the early stage of FAI. In addition, there is MRI arthrography. This technology is considered to be the “gold standard” of imaging for the diagnosis of lip and cartilage damage. It has high sensitivity, specificity, and accuracy for lip and cartilage damage.

### 2.2. Basics of 3D Reconstruction

With the development of high-tech, not only does machine vision continue to gain wider applications in the fields of robot navigation, scene reconstruction, human-computer interaction, etc., people also try to expand its application scope to new fields, such as virtual home, unmanned flying/driving, virtual fitting, 3D printing, etc.

Figure 2, shows the current application of computer vision in daily life.

Three-dimensional reconstruction technology (3D reconstruction) refers to the reconstruction of physical 3D models through relevant knowledge and technology, so as to facilitate the cognition of 3D information. There are two types of three-dimensional structure measurement methods, namely, contact and non-contact. According to the imaging principle, the non-contact method is divided into two types: active and passive. The active method requires laser or infrared and calculates the round-trip flight time or projection of light, or deformation of the pattern to obtain depth, such as laser scanning, structured light, ToF camera, etc. In the passive method, special light sources such as stereo vision technology are not required. Active technology is often limited in viewpoint and has the problem of self-occlusion. Passive technology can only rely on the existing content of the scene. Compared with active technology, its application range is limited [23].

Three-dimensional reconstruction can be divided into position estimation and normal estimation according to the different surface reconstruction methods. The position estimation technology directly estimates the position of the space surface, the technology is robust, and it is very suitable for restoring rough geometry. However, they cannot recover small-scale surface changes. The techniques for directly estimating the 3D position of the surface include not only active technologies such as laser scanning, ToF, and structured light, but also passive technologies such as passive stereo algorithms. The normal estimation technique estimates the direction of the surface given by its normal field, and integrating the normal field can restore the shape of the surface, such as shape restoration from shadows, photometric stereo vision, etc. Since the normal field is very sensitive to small changes on the surface, these techniques perform well in restoring fine structures. However, in practice, integration often introduces low-frequency deviation and noise, making these techniques less suitable for reconstructing rough geometry [24].

Although stereoscopic vision technology is relatively mature, this visual use technology also has its limitations. Its algorithm is very complex, easily interfered by environmental factors, and relies on environmental light sources, and low-light scenes perform poorly. No matter which matching method is still available, it solves the problems of occlusion, lack of texture features, and depth discontinuity [25]. Binocular stereo vision is a classic passive technology and the most commonly used stereo vision technology. Based on the triangulation principle, two images are used to measure the three-dimensional geometric structure, including multiple steps such as camera calibration and stereo matching. Binocular stereo matching can obtain a dense, high-resolution, high-precision disparity map. The structured light system has complex manufacturing process, high cost, short recognition distance, susceptibility to environmental interference, and long response time. The ToF technology can directly obtain depth information, can obtain a denser three-dimensional point cloud than structured light, and has better real-time performance. Its sensor manufacturing process is simple and small in size, has low performance and power consumption requirements, and has no dependence on the surface texture of the object. Its shortcomings are mainly that it will produce unreliable results at the edge of the field of view and the edge of the object, the resolution is relatively low, the measurement depth at short distances is missing, and there is a problem of multipath interference [26]. Therefore, based on the complementary characteristics between ToF depth camera and binocular stereo matching, the combination of ToF depth camera and binocular stereo technology can expand its scope of application and improve performance.

### 2.3. Camera Model

#### 2.3.1. Camera Model

The camera imaging process can be described by mathematical representations in projective geometry.

(1) $$\begin{array}{c} u^{\prime }=Ru+t. \end{array}$$

Assume that the three-dimensional vector *u* has undergone Euclidean transformation to obtain a new vector *u*', where *R* is a 3*∗*3 rotation vector, and *t* is a 3*∗*1 translation vector.

(2) $$\begin{array}{c} u_{2}=R_{1}u_{1}+t_{1},\\ {\text{u}}_{3}=R_{2}u_{2}+t_{2}. \end{array}$$

R1, R2 are rotation matrices, and t1, t2 are translation vectors.

It directly means that the transformation from u1 to u3 becomes

(3) $$\begin{array}{c} u_{3}=R_{2}\left(R_{1}u_{1}+t_{1}\right)+t_{2}. \end{array}$$

In order to simplify the calculation, the concept of homogeneous coordinates is introduced here. In the three-dimensional projective space, the point *Q* in homogeneous coordinates is expressed as

(4) $$\begin{array}{c} Q={\left(X,Y,\text{Z},W\right)}^{T},\\ \text{Q}\overset{\Delta }{=}\text{k}{\left(X,Y,Z,W\right)}^{T}. \end{array}$$

When *W* = 0, *Q* is the point of infinity. When W is not 0, *Q* is not a point of infinity.

(5) $$\begin{array}{c} Q^{\prime }={\left(\frac{X}{W},\frac{Y}{W},\frac{Z}{W}\right)}^{T}. \end{array}$$

That is, the homogeneous coordinates are divided by the last item at the same time. Generally, let *W* = 1.

The equation of the plane in the three-dimensional Euclidean space is expressed as

(6) $$\begin{array}{c} AX+BY+CZ+D=0. \end{array}$$

The corresponding three-dimensional projective space is expressed as

(7) $$\begin{array}{c} \text{L}={\left(A,B,C,D\right)}^{T}. \end{array}$$

On plane I:

(8) $$\begin{array}{c} Q={\left(X,Y,Z,W\right)}^{T}. \end{array}$$

It satisfies

(9) $$\begin{array}{c} {\text{L}}^{T}\cdot Q=0. \end{array}$$

Its expression in the two-dimensional projective space is

(10) $$\begin{array}{c} L={\left(a,b,c\right)}^{T}. \end{array}$$

And for any non-zero constant, *k* represents the same straight line. In the two-dimensional projective space, the necessary and sufficient conditions for the point P to be on the straight line *i* are

(11) $$\begin{array}{c} Q^{T}\cdot i=0. \end{array}$$

The intersection point of the two straight lines i1 and i2 is the outer product of the two; namely,

(12) $$\begin{array}{c} Q=i1*i2. \end{array}$$

The straight line *i* determined by Q1 and Q2 is expressed as the outer product of the two; namely,

(13) $$\begin{array}{c} i=Q1*Q2. \end{array}$$

In homogeneous coordinates, the calculation process of the camera position change becomes linear, and the mathematical expression is

(14) a'1=Rt01a1=Ta1.

Among them, the 4*∗*4 matrix *T* is called the transformation matrix. $\left(\begin{array}{c} \text{a}\\ 1 \end{array}\right)$ is the homogeneous coordinate of the camera, and a'1 is the homogeneous coordinate of the camera position after the position change.

#### 2.3.2. Small Hole Camera Model

The camera is a common device to obtain images. Through the camera, a three-dimensional scene can be projected onto a two-dimensional plane. This process can be expressed by a geometric model.

As shown in Figure 3, the small hole camera model can well express most of the existing camera models, and the basic characteristics of its imaging are that the distance is small and the distance is large [27]. The small hole camera imaging process has the following steps.

Q is a three-dimensional point, and Q′ is a point corresponding to *Q* in the camera coordinate system.

(15) $$\begin{array}{c} \left[\begin{array}{c} X_{c}\\ Y_{c}\\ Z_{c}\\ 1 \end{array}\right]=\left[\begin{array}{cc} R & t\\ 0^{T} & 1 \end{array}\right]\left[\begin{array}{c} X_{w}\\ Y_{w}\\ Z_{w}\\ 1 \end{array}\right]. \end{array}$$

Among them, *R* is the 3 X 3 rotation matrix, and *t* is the translation coordinate, which is the 3X1 vector. Both can determine the external parameters of the camera.

Then, the imaging process is

(16) $$\begin{array}{c} Z_{c}\left[\begin{array}{c} x_{u}\\ y_{u}\\ 1 \end{array}\right]=\left[\begin{array}{cccc} f & 0 & 0 & 0\\ 0 & f & 0 & 0\\ 0 & 0 & 1 & 0 \end{array}\right]\left[\begin{array}{c} X_{c}\\ Y_{c}\\ Z_{c}\\ 1 \end{array}\right]. \end{array}$$

Normally, the result of small hole imaging is an upside-down image, which will be automatically turned into an upright image during processing inside the camera. In this process, the corresponding relationship between the various quantities is

(17) $$\begin{array}{c} \left\{\begin{array}{c} {\text{x}}_{u}=\frac{gX_{c}}{Z_{c}}\\ {\text{y}}_{\text{u}}=\frac{gX_{c}}{Z_{c}} \end{array}.\right. \end{array}$$

Among them, g is the focal length. The process is

(18) $$\begin{array}{c} \left\{\begin{array}{c} \text{u}=\begin{array}{c} x_{u}\\ k \end{array}+u_{0}\\ v=\begin{array}{c} y_{u}\\ i \end{array}+v_{0}. \end{array}\right.. \end{array}$$

The focal length and the position of the principal point of the camera are called the internal parameters of the camera.

### 2.4. Beam Adjustment

When solving the three-dimensional coordinates of the characteristic points, due to factors such as noise points and calculation errors, the obtained camera parameters and three-dimensional coordinates will be deviated. This deviation will have a great impact on the final 3D reconstruction result. In order to improve the accuracy of the results, it is necessary to deal with the errors in the measurement and calculation.

The beam adjustment is the last step of SFM sparse 3D reconstruction, and it is also a very important step. Based on the internal parameters of the camera, it minimizes the reprojection error and, in the sense of nonlinear least squares, performs high-precision reconstruction of the camera parameters and the three-dimensional structure in the image [28].

## 3. Finite Element Analysis Experiment of Femoral-Acetabular Impingement (FAI) Based on Three-Dimensional Reconstruction

### 3.1. Subjects

All the hip joint anterior radiographs in the hospital were screened out, regardless of gender, aged 14–50 years old, and BMI below 28 kg/m2. According to the proposed inclusion criteria and exclusion criteria, a total of 265 patients (530 hips) were included as the research subjects.

As shown in Table 1, for the proposed inclusion and exclusion criteria, all patients in this experiment have the right to know. Without forcing the patients to conduct the experiment, the patients agreed to cooperate in the study and signed the relevant informed consent.

As shown in Table 2, for the demographic data of the study subjects, a total of 265 patients (530 hips) were included as the study subjects. In addition, 50 patients without any FAI imaging signs were selected according to the above inclusion and exclusion criteria (100 hips) as the normal group (control group).

### 3.2. Experimental Process

Figure 4 shows the research flow chart of the whole experiment. After obtaining a standard hip joint anterior view, and then selecting 100 normal hip joints without any abnormal signs, and using the range of motion of all hip joints, it was examined by double-blind method and six matching points were taken for comparison. The hip joints with PINCER-type FAI imaging signs were selected from the experimental subjects, and the range of motion of all hip joints was checked using a double-blind method. The samples were divided into five subgroups according to different imaging signs. Finally, each subgroup was analyzed. The activities of the groups were compared with those of the normal group, and the finite element analysis was carried out using three-dimensional reconstruction technology.

### 3.3. Experimental Method

#### 3.3.1. Obtaining Method of Hip Joint Orthographic Film

The three-dimensional reconstruction system was used to complete, and all the anatomical structures of the hip joint were clear; the longitudinal distance between the midpoint of the sacrococcygeal joint and the midpoint of the pubic symphysis was less than 3 cm, the lateral distance was less than 1.5 cm, and the pelvis had no obvious tilt.

#### 3.3.2. Under the Principle of Random Double-Blind

Two senior radiologists read the obtained hip joint anterior radiographs, according to the inclusion and exclusion criteria of the PINCER FAI hip joint orthographic radiographs.

As shown in Table 3, it is based on the inclusion and exclusion criteria of the PINCER-type FAI hip joint orthographic imaging signs. The four signs are associated with corresponding symptoms.

As shown in Table 4, it is based on the inclusion and exclusion criteria of the CAM-type FAI hip joint orthographic imaging signs. Among them, it was found that femoral hip impingement occurred at the early stage of hip flexion (*α* angle >40), which was more serious (*α* angle >78) and the anterior CAM deformity may cause earlier femoral hip impaction.

#### 3.3.3. Checking the Passive Range of Motion of the Hip Joint

At the same time, under the principle of random double-blind, two senior joint surgeons used the same method to check all the above-mentioned hip joint motions, measured and recorded the results with a protractor, and took two physicians to measure the motion of each hip joint.

## 4. Finite Element Analysis of Femoral-Acetabular Impingement (FAI) Based on Three-Dimensional Reconstruction

### 4.1. 3D Reconstruction System

As shown in Figure 5, the left side of the picture is the original 3D reconstruction image, and the right side is the rotated sideways image, in order to verify the effect of the proposed improved algorithm under different influencing factors, including image rotation, noise interference, and illumination changes and other influencing factors.

Figure 6 shows a traditional stereo matching SAD algorithm. This traditional algorithm is often used for image block matching. The absolute value of the difference between the corresponding values of each pixel is summed to evaluate the similarity of two image blocks.

Figure 7 shows the algorithm matching graph optimized in this paper. It can be clearly seen that the final matching points obtained by the optimized algorithm are far more than that of the traditional SAD algorithm, which shows that the matching accuracy of this algorithm is much higher than that of the traditional algorithm.

### 4.2. Algorithm Performance Analysis

As shown in Figure 8, the traditional SAD algorithm is compared with the optimized algorithm in this paper. First, three algorithms are used to detect the feature points of the image to obtain the initial matching points. Since there are a large number of mismatches in the initial matching points, it is necessary to remove the mismatched points in the initial matching points to obtain higher accuracy. It can be found from the figure that, in the first set of data, the matching accuracy of the algorithm in this paper is 59.71%, the matching accuracy of the traditional algorithm is 33.93%, the first group is 25.78% higher, the second group is 10.68% higher, and the third group is 29.98% higher. It can be seen that as the number of initial matching points is higher, the matching accuracy will be greater.

The experiment first uses the algorithm to generate sparse matching points and uses the generated matching points as the input of the PMVS algorithm to generate a denser spatial point cloud, so as to realize the three-dimensional reconstruction of the object or the environment.

As shown in Figure 9, the left side is the initial number of faces, and the right side is the final number of faces. It can be seen that when the fixed initial number of patches is the same, the final number of patches obtained by the algorithm in this chapter is 1390 less than that of the traditional SAD algorithm, but the dimension of the feature point vector proposed by the algorithm in this paper is only half of the dimension of the feature point vector of the SAD algorithm. That is, the storage requirement is reduced by 50% compared with the SAD algorithm. Although the final number of patches is reduced by nearly 13%, the result is acceptable. When the final number of patches is fixed to 10,000, the initial patch required by the algorithm in this paper is nearly 13% more than that required by the SAD algorithm, but the total storage requirement is 56.4% of the SAD algorithm.

### 4.3. Analysis of Femoral-Acetabular Impingement Sign

As shown in Figure 10, the image on the left is the comparison of the mobility of the simple cross sign and the normal group, and the image on the right is the comparison of the mobility of the simple acetabulum and the normal group. Compared with the normal group, the range of motion of the hip joints with “cross sign” on the anterior and posterior radiographs of the hip was mainly in forward flexion, internal rotation, and adduction. The results of the two groups were statistically different (*P* < 0.05). There was no significant difference in the range of motion of the hip joint in the anteroposterior view of the hip as “too deep acetabulum” compared with the normal group (*P* > 0.05).

As shown in Figure 11, the left image is a comparison of mobility between the “cross sign + deep acetabulum” group and the normal group, and the right image is a comparison of mobility between the “cross sign + deep acetabulum” group and the normal group. The main differences in the former were flexion, internal rotation, and adduction. The results of the two groups were statistically different (*P* < 0.05). The main differences in the latter are extension, internal rotation, and external rotation. The results of the two groups were statistically different (*P* < 0.05).

## 5. Conclusion

The FAI concept has been formally put forward for more than 10 years, but there are still many disputes about it. The previous research literature on FAI has many imaging indicators for its diagnosis, and it is also mentioned that the clinical symptoms of the disease are mostly pain in the groin area during flexion, adduction, and internal rotation. However, there is no clear research on the relationship between the so-called imaging signs and joint range of motion. This study focused on the influence of related imaging signs of PINCER FAI on the range of motion of the hip joint. The results proved that when there is only one FAI imaging sign, it will also affect the range of motion of the hip joint, such as the “cross sign.” In addition, the results of this study indicate that the “excessive acetabulum,” an imaging sign used to evaluate PINCER-type FAI, may not have clinical significance when it exists alone. When “posterior wall sign” exists, in addition to extension and external rotation being affected, internal rotation will also be affected; when “posterior wall sign” combined with “acetabular protrusion,” in addition to extension, internal rotation, and external rotation, internal revenue will also be affected. The disadvantage of this article is that all samples included in this study have no hip pain in daily life. Whether the hip joint with FAI imaging signs will develop osteoarthritis requires long-term follow-up. Although the 3D reconstruction process is suitable for images collected in various ways, including images obtained by image acquisition devices such as drones and consumer cameras, the requirements for image quality are still very high. In the case of poor lighting conditions, the reconstruction effect of the image is still poor. In addition, the image collected by the mobile phone is often because the image at the focal length is clear, and the other positions are very blurred, which greatly affects the solution of the parameters. For these situations, in order to get a good modeling effect, the algorithm needs to be more robust.

## Figures and Tables

**Figure 1:** Imaging examination of the hip joint.

**Figure 2:** Application of computer vision.

**Figure 3:** Schematic diagram of the small hole camera model.

**Figure 4:** Experimental flowchart.

**Figure 5:** Original image (a), rotated sideways image (b).

**Figure 6:** Traditional SAD algorithm.

**Figure 7:** The optimized algorithm.

**Figure 8:** Algorithm performance comparison.

**Figure 9:** 3D reconstruction initial number of faces (a), 3D reconstruction final number of faces (b).

**Figure 10:** Comparison of mobility between simple cross sign and normal group (a), comparison of mobility between simple acetabular deep and normal group (b).

**Figure 11:** Comparison of mobility between the “cross sign + deep acetabulum” group and the normal group (a), comparison of mobility between the “cross sign + deep acetabulum” group and the normal group (b).

**Table 1:** Inclusion criteria and exclusion criteria.

Inclusion criteria	Exclusion criteria
Age 14-50 years old	Femoral head necrosis
No gender limit	Various types of hip arthritis
Body mass index (BMI) 19–28 Kg/m2	Lumbar disc herniation
There are imaging signs of PINCER-type FAI	History of hip injury and surgery
	Inguinal hernia
	Special occupations (martial arts, dance, etc.)
	There are CAM-type FAI imaging signs

**Table 2:** Demographic data of the research subjects.

	PINCER-type sign group	Normal group
Age	32 ± 11	34 ± 9
Gender (male/female)	104/161	27/23
Body mass index (BMI)	24.1 ± 2.5	23.6 ± 1.2

**Table 3:** Signs and signs of PINCER femoral-acetabular impingement.

Cross sign	The anterior wall of the acetabulum is on the outside of the posterior wall
Deep acetabulum	The inner wall of the acetabulum overlaps with the iliac sitting line or is on its inner side
Acetabular protrusion	The inner edge of the femoral head overlaps the iliac seat line or is inside
Posterior sign	The center of the femoral head is inside the projection of the posterior wall of the acetabulum

**Table 4:** Signs and signs of CAM femoral-acetabular impingement.

Pistol-like deformity	The depression at the junction of the femoral head and neck disappears or even bulges
Femoral neck *α* angle	>40°
Femoral head and neck eccentricity	<10 mm

## Data Availability

The data that support the findings of this study are available from the corresponding author upon reasonable request.
